The article "Research on the Filtering and Classification Method of Interactive Music Education Resources Based on Neural Network" was retracted in 2023. Reasons: signs of a paper mill; suspected computer-generated content; unreliable results or conclusions; concerns about the data.

# Research on the Filtering and Classification Method of Interactive Music Education Resources Based on Neural Network

**DOI:** 10.1155/2022/5764148

**Published:** 2022-08-17

**Authors:** Biyun Xue, Ye Song

**Affiliations:** ^1^School of Marxism, School of Music and Dance, Henan Normal University, Xinxiang, Henan 453007, China; ^2^Faculty of Education, Henan Normal University, Xinxiang, Henan 453007, China

## Abstract

This work intends to classify and integrate music genres and emotions to improve the quality of music education. This work proposes a web image education resource retrieval method based on semantic network and interactive image filtering for a music education environment. It makes a judgment on these music source data and then uses these extracted feature sequences as the emotions expressed in the model of the combination of Long Short-Term Memory (LSTM) and Attention Mechanism (AM), thus judging the emotion category of music. The emotion recognition accuracy has increased after improving LSTM-AM into the BiGR-AM model. The greater the difference between emotion genres is, the easier it is to analyze the feature sequence containing emotion features, and the higher the recognition accuracy is. The classification accuracy of the excited, relieved, relaxed, and sad emotions can reach 76.5%, 71.3%, 80.8%, and 73.4%, respectively. The proposed interactive filtering method based on a Convolutional Recurrent Neural Network can effectively classify and integrate music resources to improve the quality of music education.

## 1. Introduction

The quality of teachers is a paramount social concern, especially for parents. Teachers can be grouped as academic, music, sports, and art teachers from the physical level. Their differences can be reflected in teaching ideas, methods, education background, and emotions towards students from the philosophical level. In China, the quality of rural teachers can be improved by introducing more music, sports, and art teachers, who focus more on students' emotions and psychological well-being. Some schools try to improve infrastructure and information systems but can invest pathetically due to funding difficulties. Consequently, their soft powers, such as teaching and learning evaluation systems and hardware, including experimental sites, facilities, and equipment, are lacking terribly. This has a most adverse effect on humanistic educational courses, including music education. Meanwhile, Colleges and Universities (CAUs) lack teachers and equipment to carry out music education. From the perspective of the entire music education sector, network technology greatly impacts market segmentation and the change in market patterns [1–3]. The music education model has improved alongside its industry standardization. Insiders claim that China's music education industry is moving towards digitalization and intelligence. In the future, there will be more online and offline teaching models [4, 5].

The article "Research on the Filtering and Classification Method of Interactive Music Education Resources Based on Neural Network" was retracted in 2023. Reasons: signs of a paper mill; suspected computer-generated content; unreliable results or conclusions; concerns about the data.

The online teaching model has boomed as the Chinese government further promotes education. However, it is difficult for students to retrieve the information resource online [6]. Therefore, quickly and accurately extracting Open Educational Resource (OER) from the Internet in modern music education is a key issue. Ideally, an Online Educational Platform (OEP) should provide users with simple and convenient Human-Computer Interaction (HCI) interface and recommend query requirements clearly and naturally [7–9]. Computer visualization technology utilizes computer storage and computing power to assist human observation and creativity to obtain more extensive information and interaction between people and machines.

Effective data retrieval and query are fundamental techniques in a Big Data Ecosystem (BDE), which is very arduous. A representative technology is the “magic mirror,” resembling an amplifier in reality. It can visually process and filter information to be more intuitive. Combining technology and specific knowledge, such as combining human senses and Data Mining (DM) technology, will substantially improve people's exploration and integration of information. Under this background, this work designs a kind of intelligent music teaching based on the Semantic Web and interactive image filtering technology. Semantic Web aims to build knowledge links, while interactive image filtering aims to enhance users' search intention and improve search efficiency. In addition, on this basis, a music classification system based on Convolutional Recurrent Neural Network (CRNN) is established. The system uses the Attention Mechanism (AM) to weight the music input at each time point, thereby merging and classifying the style and emotion of music, which has a certain guiding role in improving the teaching effect of music.

## 2. Materials and Methods

### 2.1. Development and Utilization of Music OER

Multimedia technologies have changed people's production and lifestyle and have been widely used. Colleges and Universities (CAUs) provide primary human resources for China's economic construction and development. In the general quality education environment, music courses impart to students the beauty of the music and improve their overall quality, thus laying a solid foundation for future development [10–12]. Applying multimedia technology in education has promoted the deepening of educational reform and injected new vitality into China's education. Therefore, it is imperative to break the conventional teaching methods and make full use of modern scientific and technological means to improve the quality of music education. Teachers and schools should know about their advantages and teaching needs and strengthen teaching-learning integration and consistency.

The article "Research on the Filtering and Classification Method of Interactive Music Education Resources Based on Neural Network" was retracted in 2023. Reasons: signs of a paper mill; suspected computer-generated content; unreliable results or conclusions; concerns about the data.

In professional teaching, nothing is more affected by the Internet than music. The music major in China is neither classical nor traditional, and not even modern. Like other subjects, the music curriculum is also dominated by classical educational concepts, which is the rationality of human cognitive construction. The new curriculum standard emphasizes the creativity and beauty of music education and its role in cultivating students' ability and humanistic spirit. With the widespread of popular culture, many educational theorists popularize music education to cater to students' psychology. This, however, has restricted the diversified development of music education [13–15]. Due to the multiculturalism need and the pluralistic society, teachers should use sufficient excellent traditional music knowledge and OES on the Internet to supplement students outside the classroom. This will appease students' antilearning psychology and classroom behaviors. Secondly, this practice has demonstrated excellent OES that can be learned on the Internet. Students no longer passively accept the popular culture. Third, such an approach can also show music students the diversity of OES.

With the rapid development of music education in China, new educational forms emerge, forming some unique educational activities. In particular, online music education can make up for offline education. However, due to the excessive dependence on teachers, it still has certain advantages in teaching experience and effect. The future development direction of music education will be the fusion of online and offline models. Online education focuses on basic theory. Offline education implements music practices, thus forming a closed loop of teaching, learning, and practice to improve the efficiency of the whole music education [16]. The comparison between online and offline music education is shown in Figure 1. By integrating and using various teaching methods, teachers break through the limitations of students' learning and expand their thoughts and horizons to acquire music knowledge and skills, from simple to deep. Gradually, it improves students' comprehensive quality. Finally, multimedia-based music education can effectively enhance the appeal of teaching. Music education guides students to learn relevant knowledge and pick up the artistic conception. Through multimedia, music can be presented from different angles so that students can experience the charm of music art.

The article "Research on the Filtering and Classification Method of Interactive Music Education Resources Based on Neural Network" was retracted in 2023. Reasons: signs of a paper mill; suspected computer-generated content; unreliable results or conclusions; concerns about the data.

Under the background that online music sparring has been passed, the standardized model has been applied to the sparring teaching of various western and national instruments, such as piano, violin, and zither, making the sparring subjects richer and catering to the diversified music education needs of users. Among them, piano education is considered to be one of the best means of early childhood music education. Thus, the piano online sparring market derived from has a market with broad growth prospects and has occupied the mainstream position in music sparring education for a long time.  Figure 2 reveals the proportion of piano sparring in online music sparring from 2015 to 2021.

### 2.2. Music Recommendation Based on Emotion Classification in Music Education

In many digital music materials, searching efficiently and quickly by computer has attracted extensive attention of scholars worldwide. Emotion-based recognition technology is a new field to realize the natural interaction between humans and machines [17–19]. The audio signal is a kind of continuous-time series different from speech signals. As an important category of audio signals, music is “a sound composed of the human voice and (or) musical instrument sound, which has semantic information, such as rhythm, melody, or harmony.” Music is a compound and unnatural sound with unimaginable human intelligence and emotional thinking ability. Many emotions and feelings with accurate word expressions can be conveyed by music, and good music works can often cause people's emotional resonance.

Music is closely related to human hearing sensation. The emotion it expresses is difficult to quantify and has strong subjectivity and uncertainty. On the one hand, this feature determines that the physical feature parameters and implementation methods used in the music retrieval technology based on emotion classification are different from the general audio classification retrieval technology. With different music forms and performances, the same song will bring different emotional experiences to the same audience. Therefore, in the music search technology based on emotion, the first thing to consider is to associate the parameters of various emotional components, such as melody, tone, and chord, with the physical characteristics of ordinary sound signals based on the emotional experience of most people. Then, the data-driven learning algorithm can classify the emotion of specific music and search the emotion according to the classification results.

In classifying music emotion, the music source should be collected first. The original data contain miscellaneous information and must be preprocessed to obtain more complex expressionists. The band characteristics with strong emotional characteristics are extracted. Here, the music source is judged first. Then, the feature sequences are used as the emotion inputs of the fusion model of Long Short-Term Memory (LSTM) and AM [20, 21]. The LSTM-AM is used to classify the music emotion to improve classification accuracy. The logical structures of LSTM and AM are given in Figures 3 and 4, respectively.

The article "Research on the Filtering and Classification Method of Interactive Music Education Resources Based on Neural Network" was retracted in 2023. Reasons: signs of a paper mill; suspected computer-generated content; unreliable results or conclusions; concerns about the data.

In the LSTM architecture in Figure 3, firstly, determine which data needs to be remembered because of its more learning value and which data needs to be abandoned because of its low correlation. Second, conduct the first round of screening for these data. It can be seen that the architecture of the LSTM model is cumbersome. The more detailed division of cell states in the neural network also produces problems such as the test of the computing power of the model. The gated loop unit is proposed to further solve this problem.

Fusing AM into LSTM can redistribute the weight of the input data once, and the input data between layers is processed for the implicit state of all time steps of the encoder. The operation process can be expressed as follows:

(1) $$\begin{array}{c} O=\text{softmax}\left(QK^{T}\right)V. \end{array}$$

In music recommendation modeling, the user's emotion is real-time, and the top k music played the most in the user's playback records in the past seven years is selected as the source set for audio feature extraction. A new feature sequence can be obtained by weighted averaging these audio feature sequences. The process of emotion-based music classification is displayed in Figure 5.

The rhythm feature extraction method of music uses the rhythm histogram to extract 16-dimensional features, such as the quantity, period, amplitude, and ratio of the four peaks. The basic frequency domain filtering model can be expressed as follows:

(2) $$\begin{array}{c} G\left(u,v\right)=H\left(u,v\right)*F\left(u,v\right). \end{array}$$

Here, *F*(*u*, *v*) is the Fourier transform of the image. *H*(*u*, *v*) represents the filter used.

The calculation of the low-pass filter reads

(3) $$\begin{array}{c} H\left(u,v\right)=1,\\ D\left(u,v\right)\leq D_{0}, \end{array}$$

(4) $$\begin{array}{c} H\left(u,v\right)=0,\\ D\left(u,v\right)>D_{0}. \end{array}$$

In equations (3) and (4), *D*_0_ is the Euclidean Distance (ED) from the pixel point to the center point of the image.

In the Latent Dirichlet Allocation (LDA) model, if the number of music topics is set to *K*, all distributions will be expanded based on *K* topics. For the spectrum document *d* of any music, the calculation of topic distribution *θ*_*d*_ reads

(5) $$\begin{array}{c} \theta_{d}=\text{Dirichlet}\left(\overset{⟶}{\alpha }\right). \end{array}$$

Here, *α* is the hyperparameter of the distribution. *K* represents a dimensional vector.

The article "Research on the Filtering and Classification Method of Interactive Music Education Resources Based on Neural Network" was retracted in 2023. Reasons: signs of a paper mill; suspected computer-generated content; unreliable results or conclusions; concerns about the data.

For any topic *k*, the calculation of word distribution *β*_*k*_ can be expressed as follows:

(6) $$\begin{array}{c} \beta_{k}=\text{Dirichlet}\left(\overset{⟶}{\eta }\right). \end{array}$$

Here, *η* is the hyperparameter of distribution. The topic number *Z*_*d*,*n*_ and the distribution of corresponding audio words *W*_*d*,*n*_ can be obtained through the topic distribution *θ*_*d*_. The specific calculation reads

(7) $$\begin{array}{c} Z_{d,n}=\text{multi}\left(\theta_{d}\right),\\ W_{d,n}=\text{multi}\left(\beta_{Z_{d,n}}\right). \end{array}$$

Gibbs sampling algorithm can solve the conditional distribution LDA. In order to do so, the expression of conditional probability $p\left(z_{i}=k|\overset{⟶}{\omega },\overset{⟶}{z}\neg_{i}\right)$ must be obtained. First, the expression of Dirichlet distribution can be simplified to obtain the following equation:

(8) $$\begin{array}{c} \text{Dirichlet}\left(\overset{⟶}{p},\overset{⟶}{\alpha }\right)=\frac{1}{\Delta \left(\overset{⟶}{\alpha }\right)}\prod_{k=1}^{K}p_{k}^{a_{k}-1}. \end{array}$$

Here, $\Delta \left(\overset{⟶}{\alpha }\right)$ is the normalization parameter.

Equation (9) calculates the conditional distribution $p\left({\overset{⟶}{z}}_{d}|\alpha \right)$ of the *d* th spectrum document of music topics in the spectrum document.

(9) $$\begin{array}{c} p\left({\overset{⟶}{z}}_{d}|\alpha \right)=\frac{\Delta \left({\overset{⟶}{n}}_{d}+\overset{⟶}{\alpha }\right)}{\Delta \left(\overset{⟶}{\alpha }\right)}. \end{array}$$

The *k* th topic in the *d* th spectrum document is expressed as *n*_*d*_^(*k*)^ and its multiple distributions can be expressed as follows:

(10) $$\begin{array}{c} {\overset{⟶}{n}}_{d}=\left(n_{d}^{\left(1\right)},n_{d}^{\left(2\right)},\ldots ,n_{d}^{\left(K\right)}\right). \end{array}$$

According to the topic conditional distribution of a spectrum, all spectrum documents' topic conditional distribution probability and the conditional distribution probability of corresponding audio words can be calculated. The specific calculation reads

(11) $$\begin{array}{c} p\left(\overset{⟶}{z}|\overset{⟶}{\alpha }\right)=\prod_{d=1}^{M}\frac{\Delta \left({\overset{⟶}{n}}_{d}+\overset{⟶}{\alpha }\right)}{\Delta \left(\overset{⟶}{\alpha }\right)},\\ p\left(\overset{⟶}{\omega }|\overset{⟶}{z},\overset{⟶}{\eta }\right)=\prod_{k=1}^{K}\frac{\Delta \left({\overset{⟶}{n}}_{k}+\overset{⟶}{\eta }\right)}{\Delta \left(\overset{⟶}{\eta }\right)}. \end{array}$$

The words generated by the music topic will not depend on a clear spectrum document. Thus, the topic distribution of music and the distribution of topic words are independent of each other.

The article "Research on the Filtering and Classification Method of Interactive Music Education Resources Based on Neural Network" was retracted in 2023. Reasons: signs of a paper mill; suspected computer-generated content; unreliable results or conclusions; concerns about the data.

### 2.3. Music Resource Classification Based on CNN

DL method can effectively overcome the defects of traditional music classification models, thus providing a new opportunity to solve this problem. The DL model enables the computer to learn to correctly recognize songs without relying on rich acoustic and music theory knowledge [22, 23]. Accordingly, a residual gated convolution structure RGLU-SE is introduced for music feature extraction by combining with channel AM. It comprises two residual gated convolution units, an SE structure, and a maximum pooling layer. On this basis, this convolution structure is used to obtain a deeper level of abstraction to classify music resources.

The human ear's perception of sound is not linear and is more sensitive to low frequency than high frequency. Therefore, it is often necessary to transform the linear spectrum into the Mel band. In the Mel filter bank, a set of the frequency spectrum can be obtained. The basic steps of this method are as follows: firstly, the time domain signal is transformed into the frequency domain by Fourier transform, and then the frequency domain signal is processed by the filter bank with the Mel frequency scale, and the Mel spectrum can be obtained. This process can be completed using the librosa library.  Figure 6 depicts the sound spectrum of four Mel songs with different genres and categories. There are obvious differences in the sound spectrum of different genres of music.

Slightly adjusting the sound quality of the music will not affect the genre of the music. However, it will change the absolute value of each sound point at a certain rate. At the same time, it can reduce the network's sensitivity to the sound intensity and improve the adaptability to various loudness audio. Suppose an audio sample generates *m* audio clips through the slicing method. The *m* audio clips will predict the music label through the model. Assuming that the number of music categories is *k*, the prediction result of the audio clip can be expressed as follows:

(12) $$\begin{array}{c} Y=\left[\begin{array}{cccc} y_{11} & y_{12} & \ldots & y_{1k}\\ y_{21} & y_{22} & \ldots & y_{2k}\\ \ldots & & & \\ y_{m1} & y_{m2} & \ldots & y_{mk} \end{array}\right]. \end{array}$$

Here, *y*_*ik*_ represents the predicted value of the *i* th music clip ton *k* music genres. Finally, the prediction probability *Y*_*k*_ of the *k* th music genre can be expressed as follows:

(13) $$\begin{array}{c} Y_{k}=\frac{\sum_{i=1}^{m}y_{ik}}{m}. \end{array}$$

The frequency component is generally large for ordinary audio signals, and it does not have periodicity. The measurement period can be measured either in the time or frequency domain. However, the periodicity of frequency-domain measurement requires that some frequency points have regular zeros or are close to zeros. Thus, it is impossible to correctly analyze the periodicity of complex signals with more frequency components and uniform power distribution. In the time domain analysis of signals, the signals can be first processed. Then, it is assumed that they are periodic and measure the frequency. The periodicity can be distinguished after analyzing the sampled signals with the periodic mean method and fixed-point analysis method.

The article "Research on the Filtering and Classification Method of Interactive Music Education Resources Based on Neural Network" was retracted in 2023. Reasons: signs of a paper mill; suspected computer-generated content; unreliable results or conclusions; concerns about the data.

Because it is difficult to convert the signal in time. It is usually converted into energy distribution in the frequency domain. The change of energy can reflect different language features. Therefore, under Hamming window, each frame must undergo a Fourier transform to obtain the energy distribution in the spectrum. In particular, Fast Fourier Transformation (FFT) can process each frame after windowing to obtain the frequency spectrum of each frame. Then, the power spectrum of audio is calculated by the modulated method.

### 2.4. Music Garbage Image-Oriented Interactive Filtering Method

There are many useless image resources in music resources, which need to be interactively filtered to obtain valuable music education resources [24, 25]. The search engine can return feature extraction and similarity calculation of the images. Then, Affinity Propagation (AP) clustering is then performed on these images, and the clustering results are hyperbolic. Afterward, interactively operations are performed on the images to click to select irrelevant categories. On this basis, the selected images are classified into “meaningless” images using the similarity criterion.

The clustering algorithm includes the following steps: (1) the number of clusters and the center of each cluster is determined. In the core space, *K* samples are selected as the cluster center. (2) In kernel space, each sample is assigned to the closest category combination according to similarity and nearest neighbor rule. (3) The calculation of the *i*th cluster dispersion matrix can be expressed as follows:

(14) $$\begin{array}{c} S_{i}=\sum_{X\in \chi_{i}}\left(X-m_{i}\right){\left(X-m_{i}\right)}^{T}. \end{array}$$

Different search engines use different technologies and return distinct image sets. Therefore, the returned images are complementary. Using multiple search engines can obtain more abundant image resources. However, many duplicate images will be generated, which must be removed. Thus, image searching first quickly finds the corresponding hash bucket through the hash index and then performs the Scale Invariant Feature Transform (SIFT) feature matching the images in the bucket to find duplicate images. The key to implementing Locality Sensitive Hashing (LSH) is to design an appropriate hash function family. Each hash function can be determined by randomly selected *a* and *b*. Common hash functions can be expressed as follows:

(15) $$\begin{array}{c} h_{a,b}\left(v\right)=\left[\frac{a\cdot v+b}{r}\right]. \end{array}$$

Here, *a* and *b* are the engineering matrix and a random number. *b* obeys the uniform distribution within [0, *r*].

The article "Research on the Filtering and Classification Method of Interactive Music Education Resources Based on Neural Network" was retracted in 2023. Reasons: signs of a paper mill; suspected computer-generated content; unreliable results or conclusions; concerns about the data.

### 2.5. Simulation Experiment Design

In terms of data set, the music downloaded from the Netease Cloud Music website is still used, which also includes song name, singer name, album name, time length, and other related data, totaling 10000 songs. Netease Cloud Music has a rich and detailed inventory of music emotions and themes. Some are built according to their own emotional status, while others create song lists according to personal interests or other customized methods. From this point of view, many songs are created by multiple users with high real-time performance. They can reflect the preferences of groups of people. Thus, these songs have a high reference value.

Music emotions are grouped as excited, relieved, relaxed, and sad emotions, with each having one or more emotional markers. The song length is no more than 6 minutes. The spectrum of the song is divided into a three-second-long segment, with each containing 56 dimensions of feature information. In the user's playback record, set the value of *k* to 10. In each training, the number of samples, learning rate, and epoch for each training in the AM is set to 120, 0.001, and 1,000. The tanh function is used as the activation function.

## 3. Results and Discussion

### 3.1. Comparison of the Effect of Music Emotion Discrimination

Respectively, 56-dimensional spectrum features are passed through the LSTM model. The 56-dimensional spectrum features are passed through the BiGRU model. The 56-dimensional spectrum features are transmitted through the BiGRU-AM model. The 56-dimensional spectrum features are transmitted through LSTM-AM. It is also compared with other common models, including Support Vector Machine (SVM) and LDA. Under different recommended models, the comparison results are plotted in Figure 7.

Apparently, after adding the music rhythm feature sequence, the newly adopted BiGRU model fully considers the time correlation of the feature sequence and strengthens the front and back connection of the feature sequence in the time sequence. The subsequent Self-Attention also strengthens the calculation ability of the model, which has a higher accuracy of music emotion discrimination and is better than the traditional neural network model. At the same time, compared with the proposed LSTM-AM, the BiGRU-AM integrates 56-dimensional features and has higher accuracy in music emotion discrimination.

The article "Research on the Filtering and Classification Method of Interactive Music Education Resources Based on Neural Network" was retracted in 2023. Reasons: signs of a paper mill; suspected computer-generated content; unreliable results or conclusions; concerns about the data.

In classifying music emotions, the diversity of emotion categories (excited, relieved, relaxed, and sad) should be considered while distinguishing emotions. The accuracy of the emotion recognition model is listed in Table 1. Emotion recognition accuracy has increased after improving the LSTM-AM into the BiGRU-AM model. The greater the difference in emotion categories, the easier it is to analyze the emotion feature sequence, and the higher the recognition accuracy is.

### 3.2. The Multitarget Detection Performance of Lightweight DL Network

This section tests the classification performance of different pooling features and their combinations in the global pooling feature aggregation layer. Three different methods are used to output the RGLU-SE stacking layer feature map, and the results are compared in Figure 8. Apparently, the aggregation of the two global pooling features gives the model higher accuracy. The accuracy of the global average pooling feature alone is higher than that of the global maximum pooling feature alone. Hence, the overall statistical information has proved to be a better comprehensive classification performance.

Four seconds, five seconds, and six seconds are selected for model classification experiments with different overlap rates. The comparison of classification accuracy of different audio segmentation overlap rates is revealed in Figure 9. According to Figure 9, the accuracy of the overlap method under three slice durations is improved compared with the overlap rate of 0%. The main reason is that the overlap method can shift the audio signal to enhance the data effect. At the same time, a 50% overlap rate has achieved the best classification performance, indicating that the appropriate overlap rate is conducive to model classification performance.

## 4. Conclusion

Music's role in ideological education does not rely on coercion but on the distinctive rhythm, charming melody, rich harmony, and beautiful timbre of music to resonate with human feelings. Therefore, music can touch the emotional center of students, awaken their hearts for art, and impact students' emotional world, ideological sentiment, and moral concepts *U*.

The article "Research on the Filtering and Classification Method of Interactive Music Education Resources Based on Neural Network" was retracted in 2023. Reasons: signs of a paper mill; suspected computer-generated content; unreliable results or conclusions; concerns about the data.

This work fully utilizes the basic signal features of music and classifies and recommends different music information by using RNN technology and AM. The proposed music classification model includes the music representation learning layer, sequence modeling, sequence feature aggregation layer, and full connection layer. Using DL to process large-scale music information helps develop and effectively process various music genres. On this basis, the sound spectrum is taken as a whole, which overcomes the difficulty of manual selection and avoids the distortion of sound signals. In this work, a music classification system based on CRNN is established. The system uses the attention mechanism to weight the music input at each time point, to merge and classify the style and emotion of music, which has a certain guiding role in improving the teaching effect of music. However, the music information may be lost in converting the sound spectrum. Future work is expected to use the sound signal of the original music as the input of the neural network and extract features. It is hoped to improve the music recognition effect of the model.

## Figures and Tables

**Figure 1:** Comparison of online and offline music education.

**Figure 2:** Proportion of piano sparring in online music sparring from 2015 to 2021.

**Figure 3:** LSTM structure.

**Figure 4:** AM structure.

**Figure 5:** Emotion-based music classification process.

**Figure 6:** Mel's music clips of songs of different genres. (a) Pop, (b) blues, (c) jazz, and (d) disco.

**Figure 7:** Comparison of music emotion discrimination results obtained from different models.

**Figure 8:** Comparison of accuracy of different pooling methods.

**Figure 9:** Comparison of accuracy of different pooling methods.

**Table 1:** Accuracy of emotion recognition model.

Recognition rate (%)	Excited	Relieve	Easily	Sad
Excited	76.5	12.4	8.5	2.6
Relieve	8.6	71.3	15.5	4.6
Relaxed	3.0	12.5	80.8	3.7
Sad	4.8	7.1	14.7	73.4

## Data Availability

The dataset used in this paper is available from the corresponding author upon request.
